The article "Assessment of the Knowledge Level of First Aid among Medical Students in Work Environment" was retracted in 2023. Reason: compromised peer review.

# Assessment of the Knowledge Level of First Aid among Medical Students in Work Environment

**DOI:** 10.1155/2022/8381819

**Published:** 2022-05-30

**Authors:** Asma Alanazi, Saad Algethami, Mohammed Alnafisah, Saoud Alhussayen, Fares Almutairi, Sultan Almureef, Maram Albalawi, Farida Habib

**Affiliations:** ^1^College of Medicine, King Saud Bin Abdulaziz University for Health Sciences (KSAU-HS), Riyadh, Saudi Arabia; ^2^King Abdullah International Medical Research Center, Riyadh, Saudi Arabia; ^3^Department of Biostatistics and Bioinformatics, King Abdullah International Medical Research Center, Riyadh, Saudi Arabia; ^4^Collage of Nursing, Minoufia University, Shibin Al Kawm, Egypt

## Abstract

First aid is one of the most important life-saving skills a health provider specifically or anybody generally must have. It can be defined as the first treatment one provides at the site of the accident to the injured person until full medical treatment is available. In some emergency situations, simple first aid can make a life-or-death difference. *Aim*. This study is designed to evaluate the knowledge of first aid among medical students at KSAU-HS in Riyadh, Saudi Arabia. *Methods*. The cross-sectional study is conducted in KSAU-HS, Riyadh, about the knowledge of first aid among medical students. A self-administered structured questionnaire is used for the purpose of data collection. The main variables are as follows: to compare the knowledge of first aid between male and female medical students, among different years of study, and identify the percentage that have knowledge of first aid. *Results*. Out of 326 students, 10 students (3.1%) scored excellent, 99 (30.4%) good, 136 (41.7%) average, 75 (23%) poor, and 6 (1.8%) very poor. *Conclusion*. The level of knowledge improved with the advancement in years, but this was not sufficient, and more training should be given to all medical students on first aid.

## 1. Introduction

What is first aid and how important is it? Well, it is an important life-saving skill a health provider specifically or anybody generally must have. One can define it as the first treatment provided at the site of the accident to the injured person until full medical treatment is available. First aid can make a life-death difference on emergencies. The Red Cross survey found that if first aid was conducted before ambulance arrives, it can prevent 59% of deaths [1–3].

Locally, a study was conducted in 2018 to evaluate the knowledge of first aid among medical students at King Saud University with a sample size of 200, 50% males and 50% females made up of 40 students (20%) from each year, 68% of students correctly answered first aid questions, with fifth-year students displaying a higher degree of knowledge. However, there were no significant differences in information between the first, second, or third-year students. The study notes that statistically there is no significant gap in first aid skills between male and female students [4–6].

The article "Assessment of the Knowledge Level of First Aid among Medical Students in Work Environment" was retracted in 2023. Reason: compromised peer review.

Likewise, Princess Norah University conducted a study in 2019 with a sample size of 1000 female students to determine the knowledge of medical students and nonmedical students about first aid skills. It was shown by the result that only 34.7% had excellent knowledge, 57.5% had medium knowledge, and 7.8% had poor first aid knowledge [7, 8]. A study was also conducted in 2019 at Taif University about the awareness, knowledge, attitudes, and practices of first aid skills among medical and nonmedical students. It was found that 56.6% of 500 participants had good first aid knowledge, while 43.4% were poor. Medical students also had a higher level of awareness than literary or other science students [9].

From a global perspective, based on a study of 152 students done at the medical college in Mangalore city, south India, in 2011, only 11% of them had previous first aid training. A total of 13% of students had good knowledge, 68.4% of students had moderate, and 17.8% of students had poor knowledge of first aid [10, 11]. An additional study carried out at Vydehi Medical College in Bangalore found that 150 medical students filled out the questionnaire, 50 from each of 5^th^ (2^nd^ year), 7^th^ (3^rd^ year), and 9^th^ terms (4^th^ year). The overall scores were as follows: 43 out of 150 students had excellent knowledge, 71 out of 150 needed improvements, 35 out of 150 had adequate knowledge, and only 1 out of 150 had poor knowledge in first aid. There was a statistically significant association between terms and level of knowledge [12–14]. Likewise, in a study on 222 final year students conducted at AIMST University, Malaysia, during June and August in 2018, majority of the students were females which accounted for approximately 63%, and the males were the rest 37%. The students included 3 different faculties with 33.3% (74) from pharmacy faculty, 32.9% (73) from dental faculty, and 33.8% (75) from medical faculty. Overall, the medical students recorded the most correctly answered questions in comparison to students from the pharmacy and dental schools, indicating that there is a significant difference in knowledge among the 3 faculties [15].

Despite of all these, first aid is a crucial skill for everyone, as anyone could face emergencies during their day. In a specific manner, junior doctors or medical students are generally expected to be able to perform basic life support skills, including cardiopulmonary resuscitation (CPR) in an emergency [16–18].

The article "Assessment of the Knowledge Level of First Aid among Medical Students in Work Environment" was retracted in 2023. Reason: compromised peer review.

In the previous studies that have been mentioned earlier, the knowledge of first aid was not as good as expected. Furthermore, this study was conducted, so that these expectations can be met and the knowledge of first aid can be evaluated. Also, no studies have been done in KSAU-HS on this topic. The contribution of study is assessing the knowledge of first aid among the medical students of KSAU-HS, Riyadh.

## 2. Methods

The study is a cross-sectional design. In a cross-sectional study, the information is collected at one point in time as the objective of the study is the assessment for knowledge and attitude; thus, a cross-sectional study is the optimum study design for this project. A self-demonstrative questionnaire-based study targets the medical college of King Saud bin Abdulaziz University of Health Sciences (KSAU-HS) in Riyadh, Saudi Arabia. KSAU-HS was founded in 2005, and it is located in King Abdulaziz Medical City, which is one of the four medical cities in Riyadh [19, 20]. It contains five colleges which are the college of medicine, science and health professions, dentistry, pharmacy, and applied medical science, with male and female college students. All students currently enrolled in the college of medicine will be included in the study population. In 2021, there are approximately 326 students practicing and studying medicine in KSAU-HS, college of medicine in Riyadh. Inclusion criteria were as follows: both male and female medical students of KSAU-HS from 3^rd^ year to 6^th^ year (batches 18, 17, 16, and 15). The questionnaire is designed in English language. It is divided into two parts: the first part includes demographic data of medical students and the second part is involved in assessing medical student's knowledge about first aid. The questionnaire will be developed and validated by experts, and the pilot study will be used to find reliability. The data will be collected by the coinvestigators in the research team. After the collection of the sheets, each sheet is coded into serial numbers using Excel 2016. The data are transferred to SAS version 9.4 for analysis. Categorical variables such as years of study and knowledge level are given as percentage and frequencies. Numerical variables (student's age and total knowledge score) are reported as mean and standard deviation. The chi-square test was used to find association between the two categorical variables (e.g. knowledge level and year of the study). All statistical tests are considered significant with *p* value less than 0.05. The proposal was submitted to the Research Unit of the College of Medicine and KAIMRC (King Abdullah International Medical Research Center) and has been approved [21]. All the participants were given an informed consent form along with the questionnaire, and the participation in the study was voluntary. The participants were free to withdraw if they wanted; also, no compensation or benefit was given to the participants. No information related to personal identification of the participants was taken. All the data collected are kept confidential, and only the research team has access to it. Anonymity of the participants is kept throughout the study and afterwards in dissemination as well.

The article "Assessment of the Knowledge Level of First Aid among Medical Students in Work Environment" was retracted in 2023. Reason: compromised peer review.

## 3. Results Section

### 3.1. Demographic Data

Data were obtained from 329 medical students (215 males and 114 females) (Figure 1) at KSAU-HS, Riyadh, Saudi Arabia, by a survey which measures the knowledge level of first aid. The survey was divided into two sections: demographic and 20 MCQs. Moreover, three surveys were removed because they were uncompleted. The scoring system was a five-point rating scale (Figure 2), the lowest was very poor, and the highest was excellent. 10 students (3.1%) scored excellent, 99 (30.4%) good, 136 (41.7%) average, 75 (23%) poor, and 6 (1.8%) very poor.

## 4. Discussion

The present cross-sectional study was carried out among 329 medical students (215 males and 114 females) at KSAU-HS, Riyadh, Saudi Arabia. We measured the level of first aid knowledge. The survey included two sections: demographic and 20 MCQs. The overall mean of the students was 21.53, while no students got a full score, and the maximum score was 38. We view this as reflecting the average knowledge of first aid. Also, the results showed a strong association with previous knowledge of first aid and the batch of students [22–24].

According to Figure 3, 214 students who had previous knowledge, certificate, and courses had higher scores in comparison to the other students. This could indicate that not only medical knowledge is sufficient to know first aid but also participating in first aid workshops, sessions, outsourcing, and attending conferences can sufficiently increase your knowledge of first aid.

According to Figure 4, we found that there is a significant difference between medical students who are in different medical school years. Batch 15 had significant higher scores than batch 18 which proves that the more advanced the students are, the more knowledge they have about first aid. 85 students from batch 15 (53 of whom are males and 32 are females) scored an overall mean of 22.69 for males and 20.63 for females. 77 students from batch 18 (50 of whom are males and 27 are females) scored an overall mean of 18.46 for males and 21.00 for females. This supports both facts that not only advancement of medical school years increases knowledge, which was indicated by the males of batches 15 and 18, but also outsourcing, attending workshops, conferences, and sessions also increase knowledge of first aid which was indicated by the females of batches 15 and 18.

The article "Assessment of the Knowledge Level of First Aid among Medical Students in Work Environment" was retracted in 2023. Reason: compromised peer review.

In comparison to previous studies, one of which is a cross-sectional study which was conducted in a medical college in Mangalore city of south India, the total participants were 152, similar to our results. 13.8% had good knowledge, 68.4% had moderate, and 17.8% had a poor level of knowledge. Another study which was conducted in undergraduate medical students of Vydehi Medical College, Bangalore, included 150 students. The overall scores were as follows: 43 out of 150 students had excellent knowledge, 71 out of 150 needed improvements, 35 out of 150 had adequate knowledge, and only 1 out of 150 had poor knowledge about first aid. Another study was conducted in 2017 at Collegium Mazovia Innovative University in Siedlce, Poland. It included 200 part-time students. 38% were very good, 51% were good, 11% were average, and 0% had lack of knowledge. In addition, a local cross-sectional study was conducted in Abha at King Khalid University. Out of 703 students, 253 were medical students, and among those medical students, 58.1% answered correctly less than 50% of questions, 20.2% answered 50–70% of the questions correctly, and 21.7% answered more than 70% of the questions.

One of the limitations during this research study was excluding batch 19 premedical students. In addition, we faced some difficulties during data collection, one of which was that the females were in a different building, and we could not reach and distribute the survey easily. Also, COVID-19 caused some difficulties in the data section because all facilities in the campus required precautionary measures.

## 5. Conclusion

First aid knowledge among medical students needs improvement. Out of 326 medical students who participated in the study, only 33.4% had good score or higher (24 or higher). The students who had a previous knowledge got a better score than those who had no knowledge before. In addition, the level of knowledge improved with the advancement in years, but this was not sufficient, and more training should be given to all medical students on first aid. We would recommend that all students either medical or nonmedical should receive mandatory first aid classes. These classes could be online sessions or in campus. Also, there should be increased awareness of first aid among the general population.

## Figures and Tables

**Figure 1:** Demographic data according to batch, gender, and measures of central tendency.

The article "Assessment of the Knowledge Level of First Aid among Medical Students in Work Environment" was retracted in 2023. Reason: compromised peer review.

**Figure 2:** Five-point rating scale.

**Figure 3:** A strong association between previous knowledge of first aid and test scores.

**Figure 4:** A strong association between the batch of participants and test scores.

## Data Availability

The data used to support the findings of this study are included within the article.
